# The Protective Mechanism of Afuresertib against Esophageal Cancer

**DOI:** 10.1155/2022/1832241

**Published:** 2022-07-14

**Authors:** Bo Min, Yan Wang, Feng Liang, Cheng-Xiang Wang, Fan Wang, Zhi Yang

**Affiliations:** ^1^Department of Thoracic Surgery, The Affiliated Huai'an Hospital of Xuzhou Medical University, The Second People's Hospital of Huai'an, Huai'an, 223002 Jiangsu, China; ^2^Department of Gastroenterology, The Affiliated Huai'an Hospital of Xuzhou Medical University, The Second People's Hospital of Huai'an, Huai'an, 223002 Jiangsu, China; ^3^Department of Gastroenterology, Jinhu County People's Hospital, Huai'an, 223600 Jiangsu, China

## Abstract

Esophageal cancer (EC) is a common malignant tumor of the digestive system. Exploring the molecular biological mechanism of EC will help to clarify its carcinogenesis mechanism, find important molecular targets in the process of carcinogenesis, and provide new ideas for the diagnosis and treatment of EC. Phosphatidylinositol-3-kinase (PI3K)/protein kinase B (Akt) signaling pathway is one of the signal transduction pathways most closely related to cell proliferation and apoptosis. The regulation of various downstream molecules affects the proliferation and growth of tumor cells. In this study, we determined the effect of different concentrations of afuresertib on cell viability by MTT assay and determined the effect of afuresertib on cell apoptosis by Annexin V-FITC/PI dual staining. Animal experiments verified the effects of afuresertib on VEGF, bFGF, and PI3K/Akt. Our results indicated that afuresertib is closely related to the survival, proliferation, and apoptosis of esophageal cancer cell lines. More importantly, we found that afuresertib could reduce tumor volume and mass in EC rats through in vivo experiments. In conclusion, afuresertib may exert its antitumor effect by inhibiting the expression of PI3K and Akt-related proteins in rat tumor tissues.

## 1. Introduction

Esophageal cancer (EC) is a common malignant tumor of the digestive system. Epidemiological survey data show that in 2018, the incidence of EC ranked seventh among malignant tumors, and the mortality rate ranked sixth [1]. China is a country with a high incidence of esophageal cancer, with new cases and deaths accounting for 53.7% and 55.7% of the global total [2]. EC is mainly divided into two subtypes, esophageal squamous cell carcinoma and esophageal adenocarcinoma, among which esophageal squamous cell carcinoma accounts for more than 95% of ES patients. EC is extremely harmful to the human body, especially in the middle and late stages of EC. Surgical treatment has high risks and many complications, which seriously affect the quality of life of patients. The 5-year survival rate for EC is less than 20% [3]. Surgery, chemotherapy, and radiation therapy are three common methods of treating EC. They have certain curative effects in inhibiting the spread of cancer cells, controlling the rate of disease progression, improving the quality of life of patients, and prolonging the survival time, but they have side effects [4–6]. Surgical resection is the method of choice for early-stage and limited-stage EC. However, due to the atypical symptoms in the early stage, most patients have metastatic cancer cells or are in the middle and advanced stages at the time of diagnosis. In addition, postoperative infection can lead to wound deterioration and increase the risk of complications [7]. Radiotherapy and chemotherapy are effective in the treatment of esophageal cancer but can cause side effects such as gastrointestinal reactions, immunosuppression, pneumonia, and esophagitis-related organic damage. It not only seriously affects the follow-up treatment effect but even accelerates the deterioration of the disease [8, 9].

The pathogenesis of EC is complex, and studies have found that it has the characteristics of multistage, multifactor, and gradual evolution. The activation of oncogenes and the inactivation of tumor suppressor genes are the basis for the carcinogenesis of esophageal cells, and this process is usually accompanied by the interaction of multiple genes [10]. Molecular biological mechanisms such as cell signal transduction, cycle regulation, differentiation, damage repair, and apoptosis are indispensable factors in the occurrence and development of malignant tumors [11]. Exploring the molecular biological mechanism of EC will help to clarify its carcinogenesis mechanism and find important molecular targets in the process of carcinogenesis, thus providing new ideas for the diagnosis and treatment of EC. Phosphatidylinositol-3-kinase (PI3K)/protein kinase B (Akt) signaling pathway is one of the signaling pathways most closely related to cell proliferation and apoptosis. It can affect the proliferation and growth of tumor cells by regulating various downstream molecules [12]. The PI3K/Akt signaling pathway is closely related to the growth and drug resistance of prostate cancer [13]. Downregulation of Circ_0000376 can inhibit the signal transduction of the PI3K/Akt pathway, thereby blocking the occurrence and development of non-small-cell lung cancer [14]. With the development of genomics research, inhibition of the PI3K/Akt pathway has been shown to inhibit tumor proliferation, but its specific mechanism in EC remains unclear [15, 16]. Afuresertib, a potent ATP-competitive and specific Akt inhibitor, has been shown to have good tumor-suppressive effects on malignant pleural mesothelioma cells, but whether it is effective against esophageal cancer cells and its mechanism of action remain unclear [17].

In this study, we explored whether afuresertib could inhibit the proliferation of esophageal cancer. The results showed that afuresertib is closely related to the survival, proliferation, and apoptosis of esophageal cancer cell lines. In vivo experiments found that afuresertib can reduce tumor volume and mass in EC rats. Afuresertib may exert its antitumor effect by inhibiting the expression of PI3K and Akt-related proteins in rat tumor tissues.

## 2. Materials and Methods

### 2.1. Laboratory Animals, Cells, and Reagents

Sixty 8-week-old female BALB/c mice were provided by the Animal Experiment Center of Beijing Institute of Life Sciences. The body weight of the rat was 200 ± 10 g. This study was approved by the Animal Ethics Committee of the Affiliated Huai'an Hospital of Xuzhou Medical University, and the rat feeding process was carried out in strict accordance with the experimental animal feeding standards. Human esophageal cancer cell line (Eca109 cells) was obtained from Procell (Wuhan, China). Afuresertib hydrochloride was provided by Selleck Chemicals, USA.

### 2.2. MTT Assay

Cell viability and growth were detected by the tetramethylazole salt colorimetric method (MTT). Cells in logarithmic growth phase were placed in a 96-well plate with 5 replicate wells for each group of cells at a cell density of 2,000 cells/well. The seeded cells were placed in a constant temperature incubator for 24 hours. Different concentrations of afuresertib (20, 10, 5, 2, 1, 0.5, 0.2, 0.1, 0.01, and 0 *μ*mol/L) were added to the cells and cultured for 24 h. 20 *μ*L of MTT solution with a concentration of 5 mg/mL was added to each well, and the medium supplemented with MTT solution was placed in a constant temperature incubator for 4 hours. Add 150 *μ*L DMSO, shake gently to mix DMSO with the cell culture medium, measure the absorbance at 450 nm with a microplate reader, and draw the cell growth inhibition curve according to the OD value.

### 2.3. Detection of Cell Growth by Plate Cloning

Cells in the logarithmic growth phase were placed in 96-well plates with 5 replicate wells per cell. The plate was placed in a constant temperature incubator for 7 days, and the medium was changed every 2-3 days for 7 days. After 7 days, cells were fixed with anhydrous methanol for 10 minutes. Methanol was removed by suction, and 1 mL of 0.005% crystal violet was added for staining. After 20 minutes of staining, crystal violet was removed by aspiration and cells were left at room temperature overnight. Clonal cells were counted the next day using a microscope.

### 2.4. Flow Cytometry

The cells in the logarithmic growth phase were placed into a 96-well plate with the density of 2,000 cells/well. Cells were treated with increasing concentrations of afuresertib for 24 h. Subsequently, 5 *μ*L of Annexin-FITC and 5 *μ*L of PI staining solution were added to cells and shaken gently until the staining solution and cell suspension are fully mixed. The mixed cell suspension was incubated in the dark for 30 min, and cell apoptosis was detected by flow cytometry within 30 min after incubation.

### 2.5. Western Blot

Cells were digested with 0.25% trypsin and washed 3 times with PBS. The RIPA buffer was added into cell pellets. The lysates were subjected to SDS-PAGE, then transferred onto a polyvinylidene difluoride (PVDF) membrane. The membrane was blocked with 5% skimmed milk for 1 hour. After washing, the membrane was incubated with the primary and secondary antibodies for 1 hour. The bands were developed with enhanced chemiluminescence (ELC) reagent and visualized by the gel imaging system (Bio-Rad, USA). The quantitation of protein expression was determined by ImageJ.

### 2.6. Real-Time PCR

The total mRNA was extracted by Trizol reagent (Invitrogen). The cDNA was synthesized using the reverse transcription kit (TaKaRa, Japan) following the instructions. The real-time PCR was performed on the ABI 7500 system (ABI, USA). The reaction system in this study was as follows: 10 *μ*L of 2 × SYBR Premix Taq II, 0.4 *μ*L of forward primer and 0.4 *μ*L of reverse primer (both at a concentration of 10 *μ*mol/L), and 2 *μ*L of cDNA template. The 2^-△△Ct^ formula was used to calculate the relative expression of the target gene with the average Ct value obtained. The experiment was repeated three times. The primers used in this study are summarized in Table 1.

### 2.7. Animal Experiments

Twelve rats were randomly selected as blank control group, and the rest were used to prepare EC models. The specific operation steps were as follows: subcutaneously inject 1 × 10^5^ Eca109 cell suspension into the axilla of the rats, and the tumor volume was 100 mm^3^ to indicate modeling success. The 48 successfully modeled rats were randomly divided into a model group, afuresertib high-dose group (20 *μ*mol/L), afuresertib medium-dose group (10 *μ*mol/L), and afuresertib low-dose group (2 *μ*mol/L) by random number method (12 in each group). The rats in each group were intervened on the next day after the successful modeling: the high-dose, medium-dose, and low-dose groups were injected with 2 mL of afuresertib with different concentrations, and the blank control group and the model group were injected with the same volume of normal saline, once a day, continuous injection for 8 weeks. After 8 weeks, the rats were anesthetized with 1% sodium pentobarbital solution (6 mL/kg) and sacrificed by cervical dislocation. The tumor was removed and placed in 4% formalin solution for fixation and placed in liquid nitrogen for freezing for future use.

### 2.8. Observation of Tumor Growth in Rats

The long diameter (*a*) and short diameter (*b*) of the rat tumor were measured with an electronic digital vernier caliper, and the tumor volume (*V*, mm^3^) was calculated (the calculation method is shown in formula 1). The tumor mass was weighed (g), and the tumor growth inhibition rate was calculated (the calculation method was shown in formula 2). Formula 1 is as follows: tumor volume = *a* × *b* × 2 × *π*/6. Formula 2 is as follows: tumor growth inhibition rate = (tumor mass of model group − tumor mass in different doses of afuresertib group)/tumor mass of model group × 100%.

### 2.9. Observation of Pathological Tissue Sections

The esophageal mucosa of normal rats and the tumor tissue of model rats were embedded to prepare tissue paraffin sections. The sections were then dehydrated using xylene and different concentration gradients of ethanol solutions (4 gradients of 70%, 80%, 90%, and 95%, each gradient 10 min). The sections were counterstained in eosin solution for 5 min, washed with water, dehydrated with absolute ethanol, and then transparentized with xylene. The slides were mounted with neutral gum, dried, and observed under a microscope.

### 2.10. Statistical Analysis

The data were analyzed using SPSS 23.0 statistical software (IBM SPSS Statistics, Armonk, NY). Quantitative data conforming to a normal distribution were expressed as mean ± standard deviation (SD), *t* test was used for comparison between two groups, analysis of variance was used for comparison between multiple groups, and LSD test was used for pairwise comparison between multiple groups. The two-sided *P* < 0.05 indicates a significant difference.

## 3. Results

### 3.1. Cell Viability Correlates with Afuresertib Concentration

The results of MTT assay showed that when the concentration of afuresertib was 0, the survival rate of Eca109 cells was 98.0 ± 1.0%. When the concentration was 2 *μ*mol/L, the cell viability was 73.0 ± 4.0%. When the concentration was 10 *μ*mol/L, the cell viability was 41.0 ± 4.0%. When the concentration was 20 *μ*mol/L, the cell viability was 22.0 ± 2.0%. As can be seen, the viability of Eca109 cells decreased with increasing concentrations of afuresertib (Figure 1).

### 3.2. Cell Proliferation Decreased with Increasing Concentration of Afuresertib

The results of plate cloning experiments showed that the proliferation of Eca109 cells decreased with the increasing concentration of afuresertib (Figure 2).

### 3.3. EC Apoptosis Rate Increased with Increasing Concentration of Afuresertib

The results of flow cytometry showed that with the increase of afuresertib concentration, the apoptosis rate of Eca109 cells increased gradually (Figure 3). It was found by WB detection that with the increase of the concentration of afuresertib, the protein levels of Bax and Caspase-3 in Eca109 cells increased, and the protein level of Bcl-2 decreased. The mRNA transcription of Bax, Bcl-2, and Caspase-3 was detected by qPCR. It was found that with the increase of afuresertib concentration, the mRNA levels of Bax and Caspase-3 in Eca109 cells increased, and the mRNA level of Bcl-2 decreased (Figures 4(a) and 4(b)).

### 3.4. Observation Results of Tumor Growth in Rats

Rats in the blank control group had no tumors, and the rats in the other groups all had mastoid tumor-like appearance with the naked eye, and the tumor formation rate was 100%. Compared with the rats in the model group, the tumor mass and volume of each group treated with afuresertib were significantly reduced (*P* < 0.05), and the effect of afuresertib was dose-dependent (Figures 5(a) and 5(b)). After calculation, the inhibition rates of afuresertib at concentrations of 2, 10, and 20 *μ*mol/L on rat tumors were 15.91 ± 4.90%, 25.59 ± 4.09%, and 36.84 ± 3.64%, respectively.

### 3.5. Effects of Afuresertib on Tumor Histopathology in EC Rats

The staining of rat tumor tissue showed that the esophageal mucosa epithelial layer of normal rats was thin, the squamous epithelial cells were tightly spaced, and there were no obvious inflammatory cell infiltration and squamous epithelial hyperplasia. In the tumor tissue of the model group, the cells were irregularly arranged, the nuclei were larger, the nucleoli were deeply stained, the blood sinuses were abundant, and the squamous cell tissue was severely hyperplastic. Compared with the rats in the model group, most of the cells in the tumor tissue of the rats in the low-dose and middle-dose afuresertib groups were lightly stained, and a small number of necrotic areas were seen, and the proliferation was weakened. Compared with the low-dose and medium-dose groups of afuresertib, the nuclei of the high-dose group were lightly stained, many necrotic areas were seen, the proliferation was significantly weakened, and there were fewer nuclei.

### 3.6. Effects of Afuresertib on VEGF and bFGF Proteins in Rat Tumor Tissue

Compared with the model group, the expressions of VEGF and bFGF proteins in the tumor tissues of the rats in each group were significantly decreased after afuresertib intervention (*P* < 0.05) and in a dose-dependent manner (Figures 6(a) and 6(b)).

### 3.7. Effects of Afuresertib on PI3K and Akt Proteins in Rat Tumor Tissue

Compared with the model group, the expression levels of PI3K, p-PI3K, Akt, and p-Akt proteins in the tumor tissues of the rats in each group were decreased in a dose-dependent manner after afuresertib intervention.

## 4. Discussion

To reveal the specific mechanism of the PI3K/Akt signaling pathway in the occurrence and development of EC, in this study, human esophageal cancer cell line Eca109 was cultured in vitro, and the cells were treated with PI3K/Akt signaling pathway inhibitor afuresertib to observe cell survival, proliferation, and apoptosis. The results showed that afuresertib can reduce the survival rate of Eca109 cells and inhibit the proliferation of Eca109 cells. At the same time, afuresertib can reduce the protein level of Bcl-2 by increasing the protein levels of Bax and Caspase-3 in Eca109 cells. Proapoptotic Bcl-2 and Bax proteins can induce programmed cell death by permeating the outer mitochondrial membrane and subsequently initiating a caspase cascade [18, 19]. Therefore, it is preliminarily identified that the PI3K/Akt signaling pathway plays an important role in the proliferation and apoptosis of esophageal cancer cells [20].

During in vivo experiments, it was found that except for the blank group, all the other groups had papillary tumor-like appearance. After intervention with afuresertib, the tumor mass and tumor volume in rats were significantly reduced in a dose-dependent manner. The above results indicate that afuresertib may have a certain inhibitory effect on EC rat tumors, and this effect was confirmed by observing the stained sections of rat tumor tissue. The staining of rat tumor tissue showed that the esophageal mucosa epithelial layer of normal rats was thin, the squamous epithelial cells were tightly spaced, and there were no obvious inflammatory cell infiltration and squamous epithelial hyperplasia. In the tumor tissue of the model group, the cells were irregularly arranged, the nuclei were larger, the nucleoli were deeply stained, the blood sinuses were abundant, and the squamous cell tissue was severely hyperplasia. Compared with the rats in the model group, most of the cells in the tumor tissue of the rats in the low-dose and middle-dose afuresertib groups were lightly stained, and a small number of necrotic areas were seen, and the proliferation was weakened. Compared with the low-dose and medium-dose groups of afuresertib, the nuclei of the high-dose group were lightly stained, many necrotic areas were seen, the proliferation was significantly weakened, and there were fewer nuclei.

Tumor growth and metastasis are closely related to tumor angiogenesis. VEGF and bFGF are important tumor angiogenesis promoters. VEGF is the hub connecting various networks of neovascularization, and it is also the most powerful and specific stimulator of vascular endothelial cell proliferation found so far and is closely related to the growth, metastasis, and prognosis of various tumors [21, 22]. bFGF is another important proangiogenic growth factor produced by tumor cells and macrophages, and it is also the first proangiogenic growth factor to be identified. bFGF not only participates in tumor angiogenesis but also promotes tumor cell growth while inhibiting tumor cell apoptosis [23, 24]. Currently, the use of anti-VEGF therapy to block angiogenesis in tumors or other pathological processes is very important, and bFGF plays an important role in this process [25, 26]. In this study, compared with the model group, the expressions of VEGF and bFGF proteins in the tumor tissues of the rats in each group were significantly decreased after afuresertib intervention in a dose-dependent manner. These results indicated that afuresertib could inhibit tumor cell growth by downregulating the expression of VEGF and bFGF proteins, thereby exerting a protective effect on rats.

Studies have shown that the PI3K/Akt signaling pathway is involved in the occurrence and development of various human cancers and is closely related to tumor growth, angiogenesis, patient prognosis, and treatment. At present, PI3K/Akt has become a research hotspot in tumor-targeted therapy [27–29]. PI3K can directly cause phosphorylation of the downstream effector molecule Akt. When the PI3K/Akt pathway is activated, the Akt phosphorylation level increases, and when the PI3K/Akt pathway is inhibited, the Akt phosphorylation level decreases [30–32]. In this study, compared with the model group, the expression levels of PI3K, p-PI3K, Akt, and p-Akt proteins in the tumor tissues of the rats in each group were decreased in a dose-dependent manner after afuresertib intervention. These results suggest that afuresertib may inhibit tumor growth by downregulating the expression of PI3K/Akt signaling pathway-related proteins.

## 5. Conclusions

In conclusion, our findings suggest that afuresertib may play a role in EC cell proliferation and apoptosis through the PI3K/Akt signaling pathway. Our study provides new ideas and insights for understanding the development of EC.

## Figures and Tables

**Figure 1:** The effect of different concentrations of afuresertib on the viability of Eca109 cells.

**Figure 2:** The effect of different concentrations of afuresertib on the OD value of Eca109 cells.

**Figure 3:** Effects of afuresertib on apoptosis of Eca109 cells. Flow cytometry with Annexin V-FITC/PI dual staining of Eca109 cells treated with increasing concentrations of afuresertib.

**Figure 4:** Expression of apoptosis-related proteins and genes in Eca109 cells. (a) Bax, Bcl-2, and Caspase-3 grayscale values. (b) Relative mRNA expression of Bax, Bcl-2, and Caspase-3.

**Figure 5:** The effect of afuresertib on the expression of VEGF and bFGF protein in rat tumor tissue. (a) Protein grayscale values. (b) Relative protein expression levels. Note: A, B, and C represent the comparison with the model group, the low-dose group, and the middle-dose group, *P* < 0.05.

**Figure 6:** The effect of afuresertib on PI3K and Akt proteins in rat tumor tissue. (a) Protein grayscale values. (b) Relative protein expression levels. Note: A, B, and C represent the comparison with the model group, the low-dose group, and the middle-dose group, *P* < 0.05.

**Table 1:** Primers used in this study.

Gene	Primer sequences (5′-3′)
Bcl-2	F: CATGTGTGTGGAGAGCGTCAAC
	R: CAGATAGGCACCCAGGGTGAT
Bax	F: TTTGCTTCAGGGTTTCATCCA
	R: CTCCATGTTACTGTCCAGTTCGT
Caspase-3	F: GGAAGCGAATCAATGGACTCTGG
	GCATCGACATCTGTACCAGACC
GAPDH	F: GGCCAAGATCATCCATGACAACT
	R: ACCAGGACATGAGCTTGACAAAGT

## Data Availability

All data were provided in the manuscript.
